The article "Empirical Analysis of Customer Risk and Corporate Financing Constraints Based on Supply Chain Networks" was published in 2022. Journal: Comput Intell Neurosci.

# Empirical Analysis of Customer Risk and Corporate Financing Constraints Based on Supply Chain Networks

**DOI:** 10.1155/2022/7984852

**Published:** 2022-09-16

**Authors:** Qun Bao, Ju-Ying Wang, Rui Xie, Zheng-Qun Cai

**Affiliations:** ^1^College of Accounting, Anhui University of Finance and Economics, Bengbu 233030, China; ^2^School of Foreign Studies, Anhui Jianzhu University, Hefei 230601, China

## Abstract

A supply chain's risk spillover effect will affect the customer's risk on the financing constraints of suppliers. This paper builds on the evaluation of customer risk by fuzzy mathematics, combines with the A-share listed companies in Shanghai and Shenzhen from 2007 to 2019 as a study sample, and empirically inspects the influence of customer risk on the level of corporate financing constraints. According to the study, it shows that the customer risk is currently at a moderate level, which will notably impair the supplier's external financing ability. This phenomenon is more remarkable when the monetary policy is tightened with fierce competition in the industry. This paper unveils the economic consequences of customer risk spillovers from a supply chain, enriches the study of the generation mechanism of corporate financing constraints, and provides investors and regulators with empirical evidence to appreciate corporate financing constraints.

## 1. Introduction

The issue of “difficult and exorbitant financing” has always been the main factor restricting China's economic growth. In 2016, President Xi Jinping, at an Economic Situation Expert Symposium, noted the following: “how to reduce corporate financing costs and mitigate financing constraints is pivotal in the supply-side reform.” Pursuant to the Report on the Work of the Government in 2019, the alleviation of financing constraints in the real economy was listed as a priority for the government. In a multilevel capital market, information asymmetry and principal-agent problems among investors, creditors, and enterprises can crucially influence financing constraints. The enterprise financing capacity notably varies with the financial conditions, governance level, and social status among enterprises. As per the study results, it proves that the enterprise's external economic environment [1], credit environment [2], internal financial characteristic information [3], governance characteristic information [4], accounting information quality [5], and other factors affect the level of corporate financing constraints. In the real scenario, corporate financing constraints are restricted by the enterprise's internal and external environment and are affected by the risk spillover effects of upstream and downstream companies in the supply chain.

The article "Empirical Analysis of Customer Risk and Corporate Financing Constraints Based on Supply Chain Networks" was published in 2022. Journal: Comput Intell Neurosci.

As an important stakeholder of enterprises' implicit contracts, customers have such a kind of interest relationship with suppliers that they will both prosper or lose. Customers will not only exert positive effect on upstream enterprises to integrate supply chains and conduct external supervision [6] but also bring the negative influence of risk transmission through supply chains [7]. If the enterprise of the customers of supply chain is faced with difficulties, the risks will result in spillover effects along the supply chain and bring uncertainty to the operation of enterprise, giving rise to the business crisis and financial crisis [8]. Therefore, the information about spillover effects, based on supply chain, will attract more investors and creditors. The existing study demonstrates that the risk information of customers will produce spillover effects to supply chains [9] and lead to the corresponding financial consequences of the enterprise [10]. Moreover, it will also affect the enterprise's trade credit [11], cash holdings [12], cost factors [13, 14], investment efficiency [15], profitability [16], and so on. Hence, will customer risk affect the level of corporate financing constraints? Clarifying this problem will assist us in appreciating the enterprise financing constraints and preventing and resolving the risks brought by supply chain cooperation.

Accordingly, this paper utilizes fuzzy mathematics to evaluate customer risk and adopts the data of listed companies from 2007 to 2019 to investigate the influence of customer risk on corporate financing constraints. Firstly, this paper evaluates customer risks on the basis of fuzzy mathematics. Secondly, it establishes an investment-cash-flow sensitivity model to examine whether the company has external financing constraints. Then, it uses 1089 groups of suppliers-customers to steadily match the company's annual data. The influence of customer risk on the financing constraints of suppliers is empirically inspected, and the heterogeneity of the relationship between the two under different monetary policy tightness and different industry competition levels is conducted.

Compared with the existing study, the incremental contributions of this paper lie with the following: firstly, it enriches the study of supply chain risk spillovers. Although the existing literature gives priority to the “predatory effect” and “support effect” among enterprises in the industry, it fails to elaborate the risk transmission mechanism between supply chain enterprises. In this paper, it deepens the influence of financial information and nonfinancial information transmitted vertically on the third-party investors and creditors based on the supply chain. Secondly, it enriches the economic consequences of customer information. Most of the existing literature explores the economic consequences of customer information as per customer concentration, customer surplus, and supplier-customer relationships, and it seldom considers the extent of the economic consequences of the customer's business crisis and financial crisis. Thirdly, it enriches the study of the influencing factors of financing constraints and further investigates the level of corporate financing constraints as per supply chain risk spillovers. The credit decision-making behavior of investors and creditors is more easily affected by the financial status of corporate customers. In this paper, it dynamically examines the influence of customer risk on the level of corporate financing constraints. Hence, the conclusion is more convincing.

The article "Empirical Analysis of Customer Risk and Corporate Financing Constraints Based on Supply Chain Networks" was published in 2022. Journal: Comput Intell Neurosci.

## 2. Theoretical Basis and Research Hypotheses

### 2.1. Customer Risk Evaluation Based on Fuzzy Mathematics

The customer risk is a significant factor that influences corporate financial decisions. The influencing factors of customer risk fall into customer external macro environment, customer financial status, customer operational risk, and customer relationship risk. There are various secondary evaluation indicators in each primary evaluation index. The construction of the customer risk evaluation index system is indicated by Table 1.

In this paper, it adopts the analytic hierarchy process (AHP) to calculate the weight of the primary indexes in the customer risk evaluation system and the secondary index weight under each primary index. In the AHP, the first step is to build a hierarchical structure model, which shall contain the objective layer, the criterion layer, and the scheme layer. In the second step, it establishes a pairwise comparison matrix, indicating the comparison of the relative importance of all factors in this layer to a certain factor in the previous layer. As for the element a_ij_ of the pairwise comparison matrix, it stands for the comparison result of the i^th^ factor relative to the j^th^ factor. In the third step, it needs to solve the feature vectors of the judgment matrix. In this paper, it adopts the square root method to calculate the approximate value of the matrix feature vectors. Firstly, the n^th^ root of the product of the elements of each row of the judgment matrix A is calculated. The formula can be seen as follows:

(1) $$\begin{array}{c} M_{i}=\sqrt[{n}]{\prod_{j=1}^{n}a_{ij.}} \end{array}$$

Then, it is normalized.

(2) $$\begin{array}{c} W_{i}=\frac{M_{i}}{\sum_{i=1}^{n}M_{i}}. \end{array}$$

It is concluded by calculating the largest eigenvalue of the judgment matrix.

(3) $$\begin{array}{c} \lambda =\overset{n}{\underset{i=1}{\sum }}\frac{{\left(Aw\right)}_{i}}{{nw}_{i}}\text{.} \end{array}$$

In the fourth step, the consistency of the judgment matrix is checked. CI is an indicator that measures the judgment matrix's deviation consistency, and the calculation formula is as follows:

(4) $$\begin{array}{c} CI=\frac{\lambda -n}{n-1}. \end{array}$$

The larger the CI, the worse the consistency of the judgment matrix. If it is, then the judgment matrix has complete conformity. CI=0, while CR represents consistency ratio, and its formula is as follows:

(5) $$\begin{array}{c} CR=\frac{CI}{RI}\text{,} \end{array}$$

where RI is the average random consistency index. If CR < 0.1, it means that it passes the consistency test.

The article "Empirical Analysis of Customer Risk and Corporate Financing Constraints Based on Supply Chain Networks" was published in 2022. Journal: Comput Intell Neurosci.

Then, calculate the comprehensive weight of each secondary indicator and sort each indicator. The results are as shown in Table 2.

Generally, the evaluation level of customer risk falls into five levels, namely, low-risk, relatively low-risk, medium-risk, relatively high-risk, and high-risk, and their risks show an increasing trend. For low-risk customers, their business environment is more stable. They have larger assets with better profitability and debt repayment capacity. They also have less operational risk. For medium-risk customers, there are certain risks in their business environment, financial status, and operation. However, they also have assets available for collateral, which can be timely settled after collection in previous transactions. For high-risk customers, their business environment is uncertain. They have a poor financial situation and credit level, and they are recognized as bad enterprises in the industry. In this paper, it utilizes the method of fuzzy comprehensive evaluation to evaluate customer risk.

In the fuzzy comprehensive evaluation, in the first step, it needs to determine the customer risk evaluation index set U.

(6) $$\begin{array}{c} U=\left\{u_{1},u_{2},\ldots ,u_{m}\right\}\text{.} \end{array}$$

In the second step, it requires to confirm customer risk evaluation level set V.

(7) $$\begin{array}{c} V=\left\{v_{1},v_{2}{,\ldots ,v}_{n}\right\}. \end{array}$$

In the third step, it needs to establish a fuzzy relationship matrix R.

(8) $$\begin{array}{c} R=\left[\begin{array}{cc} \begin{array}{cc} r_{11} & r_{12}\\ r_{21} & r_{22} \end{array} & \begin{array}{cc} \ldots & r_{1n}\\ \cdots & r_{2n} \end{array}\\ \begin{array}{cc} \vdots & \vdots \\ r_{m1} & r_{m2} \end{array} & \begin{array}{cc} \ddots & \vdots \\ \ldots & r_{mn} \end{array} \end{array}\right], \end{array}$$

where r_ij_ indicates the membership degree of customer risk to the fuzzy subset of v_i_ level in terms of index *u*_i_.

The article "Empirical Analysis of Customer Risk and Corporate Financing Constraints Based on Supply Chain Networks" was published in 2022. Journal: Comput Intell Neurosci.

In the fourth step, it requires determining the fuzzy weight vector (a_1_, a_2_,…,a_m_)for customer risk. Here, the weights obtained above using the AHP method are imported.

In the fifth step, it is to obtain the final fuzzy comprehensive evaluation model.

(9) $$\begin{array}{c} B=A\cdot R=\left(a_{1},a_{2}{,\ldots ,a}_{m}\right)\left[\begin{array}{cc} \begin{array}{cc} r_{11} & r_{12}\\ r_{21} & r_{22} \end{array} & \begin{array}{cc} \ldots & r_{1n}\\ \cdots & r_{2n} \end{array}\\ \begin{array}{cc} \vdots & \vdots \\ r_{m1} & r_{m2} \end{array} & \begin{array}{cc} \ddots & \vdots \\ \ldots & r_{mn} \end{array} \end{array}\right]=\left(b_{1},b_{2}{,\ldots ,b}_{n}\right)\text{.} \end{array}$$

Among them, *b*_i_ indicates the membership of the customer risk to the fuzzy subset of the v_j_ level as a whole.

To make the customer risk evaluation results more intuitive, in this paper, it establishes a set C to represent the evaluation results of the judges on the risk degree of each index factor that influences the customer risk.

(10) $$\begin{array}{c} C=\left\{Low\;risk,lower\;risk,me\;di\;um\;risk,higher\;risk,high\;risk\right\}=\left\{1,3,5,7,9\right\}. \end{array}$$

In this paper, it adopts the expert scoring method to determine the evaluation set for customer risk. The sorting results are indicated by Table 3.

As indicated by Table 3, it shows that the fuzzy comprehensive evaluation is conducted for each index and different risk degrees. By constructing a 13 × 5 weight judgment matrix *R*, the membership degrees of five risk level sets are finally calculated. *B* = (0.138, 0.134, 0.3, 0.256, 0.171), as indicated by Figure 1.

As illustrated in Figure 1, it intuitively proves that “medium risk” has the highest membership degree. Meanwhile, we can get V = B·C^T^ = 5.377 by calculating the evaluation score. Since 5.377 is between 5 and 7 and close to 5, we can finally judge that the evaluation result of customer risk is “medium risk.” It means, considering the factors of external macro environment, the enterprise's financial situation, operating conditions, external relations, and others, the customer company generally has certain operational risks. Its financial status and reputation level cannot be fully guaranteed, however, the probability of risk is not high. Therefore, there is some uncertainty in the expected income.

### 2.2. The Influence of Customer Risk on Corporate Financing Constraints

Pursuant to the theory of information asymmetry and principal-agent theory, in the capital market and listed companies have always seen the phenomenon of the low quality of information disclosure, and financial institutions like banks are in a disadvantageous position in the credit process. To reduce credit risk, various financial institutions, during the process of making credit decisions, will raise loan interest rates and restrict the scope of use of loan funds, thereby substantially increasing corporate financing costs and financing constraints [17, 18].

The article "Empirical Analysis of Customer Risk and Corporate Financing Constraints Based on Supply Chain Networks" was published in 2022. Journal: Comput Intell Neurosci.

Whether the information publicly disclosed by downstream customers can affect the credit decisions of creditors and investors of suppliers depends first on whether the public information is valuable to investors to evaluate corporate credit risks. Meanwhile, investors and creditors have strong information collection capabilities. Besides collecting public information, they can also obtain private customer information associated with credit risk [19]. The negative spillover influence of customer risk on supplier companies affects the credit risk of supplier companies through two aspects.

Firstly, the customer risk degree will affect their ability to perform contracts and increase the commercial credit period and bad-debt losses on accounts receivable. When the customer's operating performance declines, its ability and willingness to observe the contract decrease [20, 21]. It, in turn, affects the capital turnover efficiency of suppliers, leading to a cash flow crisis and raising credit risk. Meanwhile, customer risk will make its demand for products from upstream suppliers substantially fall off, and the company cannot transform customer resources in the short term, indicating that the company's bargaining power will decline. At this time, customers require suppliers to provide more business credit concessions terms, which further impairs the cash flow of upstream companies, so that it is detrimental to creditors and investors in evaluating the company's capacity to repay loans [22]. Furthermore, enterprises cannot open up new marketing channels. To maintain a stable supply chain relationship and sustain the supply chain's coordinated operation, the supplier enterprise decreases the risk of future sales revenue and guards against weakening the enterprise's capacity to create cash flow in the future. It provides more business credit based on risk sharing motivation to help customers overcome difficulties, which will also cause short-term cash flow crisis of enterprises and affect financing capacity [23].

Secondly, customer risk will reduce the collateral value of proprietary assets of upstream supplier relationships, so that the investors' evaluation of their credit risk can be affected. In case that a customer encounters a financial crisis, its financial risk is essentially shared by all stakeholders, and it is hard for the supplier to withdraw from the supply chain relationship. This additional risk it takes will evidently reduce the value of relationship assets [24]. Particularly with the cooperation with key customers, supplier enterprises have established a close competitive and cooperative game relationship with them and invested more proprietary assets. Once their contractual relationship is terminated, caused by customer risk in the supply chain, the proprietary assets of the relationship will be considerably depreciated, meanwhile facing high conversion costs. This makes it impossible for companies to improve their credit status and weakens credit risks by mortgaging their proprietary assets. In view of the above analysis, in this paper, it proposes the following assumptions:

**H1.**

pursuant to the supply chain risk spillover effect, the higher the customer risk, the greater the level of corporate financing constraints.

The article "Empirical Analysis of Customer Risk and Corporate Financing Constraints Based on Supply Chain Networks" was published in 2022. Journal: Comput Intell Neurosci.

### 2.3. The Regulatory Role of Monetary Policy

Monetary policy transmits market signals and affects banks' market expectations and credit decisions. It influences the financing constraints of enterprises through interest rates and credit [25]. According to the monetary policy transmission theory, from the formulation to the influence on the investment and financing of enterprises and other economic activities, the monetary policy is mainly realized through the two channels of money and credit [26]. In case it has a loose monetary policy, enterprises can increase the effective demand of the product market by stimulating the aggregate demand, thus enhancing the profitability of the enterprise [27]. The weakening of profitability decreases the business operation risk of enterprises because of the negative amplification effect caused by customer risk spillover. Meanwhile, under a loose monetary policy, it can increase the total supply of bank credit and enhance the enthusiasm of bank loans. Even though the enterprise's business conditions are affected by customer risk contagion, the conditions of bank loans will be relaxed, which, in turn, can improve the external financing environment of enterprises and increase the financing ability [28]. In view of the above analysis, in this paper, it proposes the following assumptions:

**H2.**

loose monetary policy can alleviate the deterioration of customer risk on corporate financing constraints

### 2.4. The Regulating Effect of Industry Competitiveness

In the capital market, the industry competitions will have a differentiated effect on the main business through the “predatory effect” opportunistic behavior. More precisely, when the enterprise industry is highly competitive, the “predatory behavior” of other competitors in the industry will create operational uncertainty risks [29]. The enterprise customer risk is relatively high. Based on the risk contagion of the supply chain, the competitive position of supplier companies is substantially decreased. At this time, provided that the company industry is highly competitive, the situation it faces is even more severe, and the “predatory behavior” of other companies in the industry will have greater impact [30, 31]. Meanwhile, highly competitive industries will face the disadvantages of small market share, slow growth, and fewer investment opportunities. Financial institutions like investors and creditors have higher requirements when making credit decisions, which notably increase the level of financing constraints for suppliers [32]. In view of the above analysis, in this paper, it proposes the following assumptions:

**H3.**

the higher the level of competition in the industry, the worse the impact of customer risk on the financing constraints of enterprises.

The article "Empirical Analysis of Customer Risk and Corporate Financing Constraints Based on Supply Chain Networks" was published in 2022. Journal: Comput Intell Neurosci.

## 3. Research Design

### 3.1. Data and Sample

In this paper, it takes the panel data of Shanghai and Shenzhen A-share listed companies from 2007 to 2019 as the initial sample and process the obtained samples as follows: (1) it eliminates the listed companies in the ST and financial industries. (2) Delete the companies whose top five customers fail to disclose their sales proportion. (3) The samples with missing study data are removed. (4) To reduce the influence of extreme values on the regression results, in this paper, the authors perform a winsorization of 1% up and down for all continuous variables. In this paper, the data come from companies whose suppliers and customers are both listed companies, which have completed the annual matching data of suppliers and customers. Customer-related data were collected manually, and other data were derived from the CSMAR database. After the above screening, it ended up acquiring1089 groups of supplier-customer matching data.

### 3.2. Definition of Variables and Model Setting

#### 3.2.1. Explained Variables

Financing constraints (invest): currently, there is no unified conclusion about the measurement of corporate financing constraints. Existing research measures financing constraints from three categories. Use enterprise characteristics to establish KZ, SA, WWS, and other indices: the cash holdings-cash flow sensitivity model; investment-cash flow sensitivity model. Fazzari and Peters [33] argued that the transaction cost caused by the problem of information asymmetry led to an increase in the external financing cost of enterprises, making the enterprises with poor financing ability more dependent on internal capital investment. Accordingly, they believed that the fluctuation of investment on cash flow notably influenced the cash flow. The higher the “sensitivity,” the greater the sensitivity coefficient of cash flow (CashFlow), indicating that the company is more dependent on internal capital investment, which, in turn, indicates that the company faces a higher level of external financing constraints, and its value is equal to net cash flows from operating activities divided by total assets. Based on the above analysis, in this paper, it selects the investment-cash flow sensitivity model to measure the level of financing constraints, and the level of corporate capital expenditure (invest) as the explained variable, whose value is equal to the cash paid for the purchase and construction of fixed assets, intangible assets, and other long-term assets divided by total assets.

The article "Empirical Analysis of Customer Risk and Corporate Financing Constraints Based on Supply Chain Networks" was published in 2022. Journal: Comput Intell Neurosci.

#### 3.2.2. Explanatory Variables

Customer risk (risk): there are many models for measuring the level of enterprise risk. The existing study on its measurement indicators contains the following: *Z* index, earnings volatility, stock return volatility, asset-liability ratio, and leverage coefficient, among which earnings volatility is the most commonly used indicator to measure corporate risk. In this paper, it learns from the research of Liu Xing [34] and adopts the volatility of return on assets (ROA) to measure the level of corporate risk. The greater the volatility of this indicator, the higher the corporate risk. Learning from the study of Coles [35], it utilized the rolling year method to calculate the standard deviation of the stock returns (*r*_i_) of the sample companies in each period with every 5 years as an observation period. The calculation process is as follows:

(11) $$\begin{array}{c} risk=\sqrt{\frac{1}{N-1}\overset{N}{\underset{n=1}{\sum }}\left(ADJ_{-}ROA_{in}-\frac{1}{N}\overset{N}{\underset{n=1}{\sum }}ADJ_{-}ROA_{in}{)}^{2}\right.},N=5, \end{array}$$

where ADJ_−_ROA_in_=ROA_in_ − 1/X∑_K=1_^X^ROA_kn_.

#### 3.2.3. Control Variable

In this paper, the control variables fall into the supplier corporate governance level, operation level, and customer level. The variables contain corporate growth (growth), corporate age (age), return on assets (ROA), shareholding ratio of the largest shareholder (hold), change in short-term current liabilities (Std), management shareholding (Msh), customer age (KHAge), and return on customer assets (KHROA). They also contain monetary policy (MP) and industry competitiveness (HHI)-regulated variables, controlling for the year and the industry. The calculation method of the variables is indicated by Table 4.

The article "Empirical Analysis of Customer Risk and Corporate Financing Constraints Based on Supply Chain Networks" was published in 2022. Journal: Comput Intell Neurosci.

#### 3.2.4. Model Specification

It adopts the basic model (12) of the investment-cash flow sensitivity model to measure the level of financing constraints.

(12) $$\begin{array}{c} {\left(\frac{I}{K}\right)}_{\text{it}}=f{\left(\frac{X}{K}\right)}_{\text{it}}+g{\left(\frac{\text{CF}}{K}\right)}_{\text{it}}{+\varepsilon }_{\text{it}}\text{.} \end{array}$$

Among them, K indicates capital stock, I indicates investment expenditure, CF refers to cash flow from operating activities, *X* stands for a variable that theoretically determines the investment demand of an enterprise, and g refers to the sensitivity of enterprise investment to fluctuations in internal cash flow. Drawing on the study of Wan Liangyong [36], it adopts the investment-cash flow sensitivity model to verify the existence of external financing constraints of enterprises, in which sensitivity coefficient is used as the factor of financing constraints. Measure the indicators and build the model (13) as follows:

(13) $$\begin{array}{c} {\text{Invest}}_{\text{it}}{=\alpha }_{0}{+\alpha }_{1}{\text{CashFlow}}_{\text{it}}{+\alpha }_{2}{\text{Growth}}_{\text{it}}{+\alpha }_{3}{\text{Age}}_{\text{it}}{+\alpha }_{4}{\text{ROA}}_{\text{it}}{+\alpha }_{5}{\text{Hold}}_{\text{it}}{+\alpha }_{6}{\text{Std}}_{\text{it}}\\ {+\alpha }_{7}{\text{Msh}}_{\text{it}}+\sum \text{Industry}+\sum \text{year}{+\varepsilon }_{\text{it}}\text{.} \end{array}$$

To study the relationship between customer risk and financing constraints, namely, hypothesis H1, we add customer risk factor to build model (13) and add customer characteristic factors like customer age (KHAge) and return on customer assets (KHROA) to build a model (14).

(14) $$\begin{array}{c} {\text{Invest}}_{\text{it}}{=\alpha }_{0}{+\alpha }_{1}{\text{CashFlow}}_{\text{it}}{+\alpha }_{2}{\text{CashFlow}}_{\text{it}}{*\text{risk}}_{\text{it}}{+\alpha }_{3}{\text{risk}}_{\text{it}}{+\alpha }_{4}{\text{Growth}}_{\text{it}}{+\alpha }_{5}{\text{Age}}_{\text{it}}\\ {+\alpha }_{6}{\text{ROA}}_{\text{it}}{+\alpha }_{7}{\text{Hold}}_{\text{it}}{+\alpha }_{8}{\text{Std}}_{\text{it}}{+\alpha }_{9}{\text{Msh}}_{\text{it}}{+\alpha }_{10}{\text{KHAge}}_{\text{it}}{+\alpha }_{11}{\text{KHROA}}_{\text{it}}\\ +\sum \text{Industry}+\sum \text{year}{+\varepsilon }_{\text{it}}\text{.} \end{array}$$

Considering the relationship among customer risk, monetary policy (industry competitiveness), and financing constraint, we verify the intermediary role of monetary policy (industry competitiveness) between customer risk and financing constraint, namely, hypothesis H2 and H3. On the basis of model (14), we construct model (15) using *X* variables, where *X* denotes monetary policy (MP) and Herfindal Hirschman index (HHI).

(15) $$\begin{array}{c} \text{Inves}t_{\text{it}}=\alpha_{0}+\alpha_{1}\text{CashFlo}w_{\text{it}}+\alpha_{2}\text{CashFlo}w_{\text{it}}*\text{ris}k_{\text{it}}+\alpha_{3}\text{ris}k_{\text{it}}+\alpha_{4}\text{CashFlo}w_{\text{it}}*\text{ris}k_{\text{it}}*X\\ +\alpha_{5}X+\alpha_{6}Growth_{it}+\alpha_{7}Age_{it}+\alpha_{8}ROA_{it}+\alpha_{9}Hold_{it}+\alpha_{10}Std_{it}+\alpha_{11}Msh_{it}\\ +\alpha_{12}KHAge_{it}+\alpha_{13}KHROA_{it}+\sum Industry+\sum year+\varepsilon_{it}\text{.} \end{array}$$

In formulas (12)–(15), *α* refers to the coefficient value, *ε* means the residual item, *i* represents different enterprises, *t* indicates the year, and the coefficient *α*_1_ of CashFlow is the investment-cash flow sensitivity.

The article "Empirical Analysis of Customer Risk and Corporate Financing Constraints Based on Supply Chain Networks" was published in 2022. Journal: Comput Intell Neurosci.

## 4. Empirical Analysis and Results

### 4.1. Descriptive Statistics

The full-sample descriptive statistics of each variable are indicated in Table 5. The maximum value of Invest is 0.2378, the mean value is 0.0564, and the minimum value is 0.0003, which indicates that there exist differences in the capital expenditures of listed enterprises. The mean value of operating cash flow (CashFlow) reaches 0.0399, which represents that annual operating cash flow accounts for 3.99% of total assets. The average value of customer risk reaches 0.0428, which indicates that 4.28% of business customers face high risk. It can be seen that there are, as a whole, fewer business customers with high risk.

### 4.2. Regression Results and Interpretation

#### 4.2.1. Investment-Cash-Flow Sensitivity Model Regression Results

According to the result of column (1) in Table 6, it proves that the coefficient of capital expenditure and cash flow from operating activities is 0.0832, which is significantly positive at the 1% level, indicating that Shanghai and Shenzhen A-share listed companies generally have external financing constraints. The reason is that when corporate financing is blocked, to maintain corporate scale and enhance operating performance, companies generally choose to extract some funds from internal cash flow for investment. Considering the above analysis, the investment-cash flow sensitivity coefficient is notably positive.

#### 4.2.2. The Impact of Customer Risk on Corporate Financing Constraints

In Column (2) of Table 6, it displays the regression result of the full-sample customer risk and corporate financing constraints. Among them, the coefficient before the interaction term between customer risk and operating cash flow represents the degree to which the investment-cash-flow sensitivity is affected by the enterprise customer risk. Provided that the coefficient of the interaction term is obviously positive, the higher the customer risk will aggravate the level of external financing constraints, the larger the coefficient, and the greater the impact. According to the result of column (2) in Table 6, it shows that the coefficient of the interaction term between customer risk and cash flow from operating activities is notably positive at the 5% level. The parameter estimate of cash flow from operating activities to capital expenditure reaches 0.0690, and at 5% is notably positive at the level. It shows that the higher the customer risk, the higher the level of enterprise financing constraints. Hence, hypothesis H1 has been verified.

The article "Empirical Analysis of Customer Risk and Corporate Financing Constraints Based on Supply Chain Networks" was published in 2022. Journal: Comput Intell Neurosci.

#### 4.2.3. The Influence of Monetary Policy and Industry Competitiveness on the Relationship between Customer Risk and Corporate Financing Constraints

Pursuant to the regression results in Table 7, it proves that, after the introduction of monetary policy and industry competitiveness, the coefficient of interaction among customer risk, monetary policy, and operating cash flow is −0.2433, which is significantly negative at the 10% level. It shows that compared with tight monetary policy, the level of financing constraints when monetary policy is loose is less affected by corporate customer risk. The coefficient of interaction item between customer risk, industry competitiveness, and capital expenditure reaches −6.6113, which is notably negative at the 10% level. It indicates that customer risk positively influences financing constraints compared to less competitive companies in the industry. The effect of the directional influence on the enterprises with a high degree of competition in the industry is more significant. Hence, the hypothesis H2 and H3 are supported.

### 4.3. Robustness Test

#### 4.3.1. Replace the Explained Variable

Drawing on the study of Hong Jinming and Lin Runyu et al., the observation period is defined as from year *t* to year *t*+2 to redefine the level of customer risk taking and substitute it into the model (14). Upon inspection, the replaced customer risk makes the regression result consistent with the previous text. Hence, it is concluded to be robust. The regression results in column (1) of Table 8 are as follows:

#### 4.3.2. Other Sensitivity Test

To prevent the omitted variable from causing a positive correlation between customer risk and the level of suppliers' external financing constraints, the model contains the size of the company (Size), the concurrent position of chairman and General Manager (Dual), the size of the Board of Directors (Board), and the ratio of tangible assets (PPE). Equal variables are used as control variables, and the regression results are indicated by column (2) in Table 8. Furthermore, it only considers that the manufacturing industry is with the industries other than the manufacturing industry being excluded, and the regression results are listed in Column (1) of Table 9. To prevent the influence of the privatization information of state-controlled enterprises, in this paper, it selects a sample of nonstate-owned enterprises to perform basic regression again. The empirical results are indicated by column (2) of Table 9. The above regression results are consistent with the previous text. Hence, it is concluded to be robust.

The article "Empirical Analysis of Customer Risk and Corporate Financing Constraints Based on Supply Chain Networks" was published in 2022. Journal: Comput Intell Neurosci.

#### 4.3.3. Alternate Models

The measurement of financing constraints in existing research is not uniform, and the use of SA index is more common. In this paper, it draws on the methods of HadLock and Pierce [37] to construct the SA index, SA = −0.737*∗*Size + 0.043Size^2^−0.04*∗*Age, in which, Size refers to the scale of the enterprise, Age means the year of establishment, and the absolute value of SA is used to measure the financing constraint (FC). The larger the absolute value of SA, the higher the level of corporate financing constraints. Moreover, given the high volatility of China's stock market, the stock return volatility index (CRT) can be used to measure customer risk. Meanwhile, control variables that may affect financing constraints are added to the model, and the model (16) is constructed as follows:

(16) $$\begin{array}{c} FC_{it}=\alpha_{0}+\alpha_{1}CRT_{it}+\alpha_{2}CashFlow_{it}+\alpha_{3}Age_{it}+\alpha_{4}Size_{it}++\alpha_{5}PPE_{it}++\alpha_{6}Lev_{it}\\ +\alpha_{7}Hold_{it}+\alpha_{8}Msh_{it}+\alpha_{9}ROA_{it}+\alpha_{10}Growth_{it}+\alpha_{11}Dual_{it}+\alpha_{12}KHROA_{it}\\ +\alpha_{12}KHAge_{it}+\sum Industry+\sum year+\varepsilon_{it}\text{.} \end{array}$$

The regression results are given in Table 10. The coefficient of CRT is notably positive, which means that the higher the customer risk, the greater the level of corporate financing constraints. It is in conformity with the previous text. Hence, it is concluded to be robust.

#### 4.3.4. Endogeneity

*(1) Two-stage least squares method*: based on the previous test, it is proved that customer risk affects the level of enterprise's external financing constraints, and corporate financing capacity will also restrict the conduct of customer risk activities. Therefore, it can adopt the instrumental variable method to alleviate the endogeneity problem caused by reverse causality. In this paper, it utilizes the two-stage least squares method, draws on the study of Miao Miao and Liao Shiyu (2020) [38], and introduces a one-phase lag (L. risk) and managerial overconfidence (OC) of corporate customers as the instrumental variables of customer risk to further test model (14). Among them, the overconfidence of managers affects the level of risk taking, and the indicator of overconfidence of customer managers fails to directly affect the level of suppliers' external financing constraints to meet the exogenous requirements. It adopts the personal characteristics of general managers to construct a measure of managerial overconfidence. See Tables 11 and 12 for regression result. As shown in column (1) and column (2), in the regression results of the first stage, the significance levels of L. risk and OC of the first-stage regression and L. risk*∗*CashFlow and OC*∗*CashFlow of the second-stage exceed 5%, and the F statistic values of the two regressions in the first stage exceed 10. It can indicate that there is no weak instrumental variable problem. As indicated by column (3), the variable risk*∗*CashFlow has a positive and significant sign, which means that the conclusion is still robust after using instrumental variables to deal with possible endogeneity problems. It is still concluded to be robust.

*(2) Heckman two-stage.* In this study, the sample corresponding to customer risk may not be randomly selected; however, it is rationally selected. There may be endogeneity problems caused by sample bias and self-selection between customer risk and corporate financing constraints. To this end, in this paper, it adopts Heckman two-stage regression to test again.

The article "Empirical Analysis of Customer Risk and Corporate Financing Constraints Based on Supply Chain Networks" was published in 2022. Journal: Comput Intell Neurosci.

In the first stage, the customer risk is transformed into a dummy variable with the average value as the demarcation point. The value above the average value of risk taking is 1, and the value below the average value is 0. Based on the study of Zhang Xin et al. [39], the size of the enterprise, the asset-liability ratio Lev, the return on assets ROA, the age of establishment Age, and the growth of the enterprise are selected as the main influencing factors of the risk taking level, and the first-stage Probit model (17) is constructed as follows:

(17) $$\begin{array}{c} risk_{it}=\alpha_{0}+\alpha_{1}Size_{it}+\alpha_{2}Lev_{it}+\alpha_{3}ROA_{it}+\alpha_{4}Age_{it}+\alpha_{5}Growth_{it}+\sum In\;du\;stry+\sum year+\varepsilon_{it}. \end{array}$$

It obtains the inverse Mills ratio (IMR) by performing the Probit regression on model (17), substituting it into model (14) as a control variable, and reregressing to test the previous hypothesis. Pursuant to the regression result, it proves that the IMR coefficient of the second-stage regression is not notable and the coefficient of risk*∗*CashFlow is still significantly positive, indicating that the problem of sample self-selection in this paper is not serious, and the conclusion is robust.

The article "Empirical Analysis of Customer Risk and Corporate Financing Constraints Based on Supply Chain Networks" was published in 2022. Journal: Comput Intell Neurosci.

## 5. Conclusions and Suggestions

On the basis of the evaluation of customer risk by fuzzy mathematics, in this paper, it adopts the Shanghai and Shenzhen A-share listed companies from 2007 to 2019 as a study sample to empirically test the impact of customer risk on the level of corporate financing constraints. It also investigates the heterogeneous effects of monetary policy and industry competitiveness on the relationship between them. Pursuant to the research result, it shows that customer risk is currently at a moderate level. Based on the spillover effect of supply chain risk, customer risk will increase the level of external financing constraints for suppliers. It is because customer risks will reduce their ability to perform contracts and the mortgage value of proprietary assets of the relationship. Buyers and sellers in the same supply chain are often a community of interests that “prosper, lose, and are mutually dependent,” and it is hard for suppliers to break away from the supply chain. The information publicly disclosed by downstream customers can affect the credit decisions of creditors and investors of suppliers. Investors and creditors have strong information collection capabilities. Besides collecting public information, they can also obtain private information about customers associated with credit risk. A loose monetary policy will alleviate the problem of the external financing constraints of suppliers caused by customer risks. It is because macro monetary policy restricts the price of bank credit assets, thereby causing systemic changes in the credit market. There are relatively few financing channels for listed companies in China. Most companies conduct financing activities through the banks. When the monetary policy is loose, companies are less affected by customer risks. Hence, it is easier to obtain bank credit resources. In the event that the industry is highly competitive, it will enlarge the negative spillover effect of customer risks on supplier companies and reduce corporate financing capabilities. It is because supply chain risk spillovers affect the business performance of suppliers. Provided that the industry competition is fierce at this time, companies will be affected by the same industry. The predatory behavior of other companies is more serious, and creditors and investors will increase financing conditions as per this information.

To further activate the information transmission and financing market in the supply chain, this paper, pursuant to the above conclusions, puts forward the following suggestions: firstly, when making financing decisions, enterprises should focus on the macroeconomic policies, internal corporate governance structure, and the impact of public information and private information between affiliated enterprises, especially upstream and downstream enterprises, because suppliers and customers restrict an enterprise's production and business activities. Secondly, in case it witnesses the tightening of monetary policy and fierce industry competitiveness, enterprises are less dependent on customer resources. Provided that the customers encounter risks at this time, the negative spillover effect of customer risks will be magnified, which will affect the credit decisions of investors and creditors. Finally, enterprises should fully exert their supervisory role and governance mechanism to curb the adverse effects caused by the financial and nonfinancial information of downstream customers. Meanwhile, the government shall unceasingly improve the capital market credit system, enhance the transparency of market information, and ease corporate financing constraints, thereby creating a good business environment.

The article "Empirical Analysis of Customer Risk and Corporate Financing Constraints Based on Supply Chain Networks" was published in 2022. Journal: Comput Intell Neurosci.

## Figures and Tables

**Figure 1:** Judgment of the result of risk level membership degree.

**Table 1:** Customer risk evaluation index system.

Objective layer	Primary evaluation index	Secondary evaluation index	Secondary evaluation index description
Customer risk	Customer external macro environment	Economic policy uncertainty	The degree of economic policy uncertainty in the province where the customer is located
		Industry competition environment	The competition level in the customer's industry
		Regional legal environment	The legal environment of the province where the customer is located
	Customer's financial status	Profitability	Customer business profitability, measured by earnings per share
		Solvency	The solvency of the customer enterprise, measured by the asset-liability ratio
		Operational capability	The operating capacity of the customer enterprise, measured by the total asset turnover ratio
		Development capacity	The development capacity of the customer's enterprise, measured by the revenue growth rate
	Customer's operational risk	Senior executives	Working age of senior executives
		The situation that the company is regulated	The situation that the company is punished or inquired
		Company's internal control	The effectiveness of the company's internal control measured by the internal control index
		Operational stability	Earnings volatility, measured by ROA volatility
	Customer relationship risk	Relationship investment	Whether there are relationship investments between customers
		Relational risk	Dependence on customers, measured by customer concentration

The article "Empirical Analysis of Customer Risk and Corporate Financing Constraints Based on Supply Chain Networks" was published in 2022. Journal: Comput Intell Neurosci.

**Table 2:** Customer risk evaluation index and its weights.

Objective layer	Primary evaluation index	Weight	Secondary evaluation index	Weight	Comprehensive weight	Sort
Customer risk	Customer external macro environment	0.1858	Economic policy uncertainty	0.2809	0.0522	11
			Industry competition environment	0.4140	0.0769	8
			Regional legal environment	0.3051	0.0567	10
	Customer's financial status	0.3759	Profitability	0.2929	0.1101	1
			Solvency	0.2609	0.0981	3
			Operational capability	0.2583	0.0971	4
			Development capacity	0.1879	0.0706	9
	Customer's operational risk	0.2652	Senior executives	0.1208	0.0320	13
			The situation that the company is regulated	0.1726	0.0458	12
			Company's internal control	0.3241	0.0860	6
			Operational stability	0.3825	0.1014	2
	Customer relationship risk	0.1731	Relationship investment	0.4568	0.0791	7
			Relational risk	0.5432	0.0940	5

**Table 3:** Customer risk evaluation sets.

Objective layer	Criterion layer	Index layer	Evaluation sets				
	Primary evaluation index	Secondary evaluation index	1	3	5	7	9
Customer risk	Customer external macro environment	Economic policy uncertainty	1	2	5	2	0
		Industry competition environment	1	3	4	0	2
		Regional legal environment	1	3	4	1	1
	Customer's financial status	Profitability	0	2	3	4	1
		Solvency	0	1	5	1	3
		Operational capability	1	1	4	3	1
		Development capacity	3	2	4	1	0
	Customer's operational risk	Senior executives	3	2	3	1	1
		The situation that the company is regulated	0	1	7	2	0
		Company's internal control	0	2	6	2	0
		Operational stability	1	1	3	3	2
	Customer relationship risk	Relationship investment	3	1	4	2	0
		Relational risk	1	2	5	1	1

**Table 4:** Summary table of variable definition 1.

Variable name	Symbols	Calculation method
Total assets level	Invest	Total cashes/assets paid for construction of fixed assets, intangible assets, and other long-term assets
Customer risk	Risk	Volatility of return on assets
Operating cash flows	CashFlow	Operating activities net cash flow/total assets
Growth	Growth	(Operating income at the end of the period–operating income at the beginning of the period)/operating income at the end of the period
Age of establishment	Age	The natural logarithm of the age of establishment + 1
Return on assets	ROA	Net income/total assets
Shareholding ratio of the largest shareholder	Hold	Number of shares held by the largest shareholder/total number of shares
Changes in short-term current liabilities	Std	(Short-term current liabilities in year *t−*short-term current liabilities in year t-1)/total assets in year t
Management shareholding	Msh	Number of shares held by management/total shares
Customer's age	KHAge	The natural logarithm of the customer's establishment year + 1
Return on customer assets	KHROA	Customers net income/total assets
Monetary policy	MP	M2 growth rate–GDP growth rate–CPI growth rate
Industrial competitiveness	HHI	Herfindahl–Hirschman index
Industry dummy	Industry	Sector
Year virtual variable	year	Year

The article "Empirical Analysis of Customer Risk and Corporate Financing Constraints Based on Supply Chain Networks" was published in 2022. Journal: Comput Intell Neurosci.

**Table 5:** Descriptive statistics.

Variable	N	Min	Max	Mean	P50	Sd
Invest	1089	0.0003	0.2378	0.0564	0.0421	0.0500
Cash flow	1089	−0.1541	0.2137	0.0399	0.0385	0.0661
Risk	1089	0.0016	0.2502	0.0428	0.0183	0.0655
Growth	1089	−0.9327	2.1035	0.1066	0.0962	0.4388
Age	1089	1.0986	3.4340	2.6837	2.7726	0.4281
ROA	1089	−0.2848	0.1717	0.0384	0.0398	0.0598
Hold	1089	0.1047	0.7713	0.3629	0.3393	0.1532
Std	1089	−3.6152	0.3330	−0.0837	0.0260	0.5541
Msh	1089	≤0.001	0.6923	0.1415	0.0019	0.2110
KHAge	1089	1.6094	3.4340	2.7566	2.8332	0.3586
KHROA	1089	−0.0841	0.1783	0.0438	0.0382	0.0435

**Table 6:** Regression results of customer risk and corporate financing constraints.

	(1)	(2)
	Invest	Invest
Cash flow	0.0832^*∗∗∗*^	0.0690^*∗∗*^
	(20.16)	(2.48)

Risk		0.0353
		(1.50)

Risk*∗*CashFlow		0.8925^*∗∗*^
		(2.27)

Hold	0.0027	0.0203^*∗∗*^
	(1.41)	(2.06)

Std	0.0036^*∗∗∗*^	0.0096^*∗∗∗*^
	(6.35)	(3.30)

Msh	0.0253^*∗∗∗*^	0.0347^*∗∗∗*^
	(16.59)	(4.75)

ROA	0.0417^*∗∗∗*^	0.0520^*∗∗*^
	(8.43)	(2.03)

Growth	0.0007^*∗*^	−0.0020
	(1.85)	(−0.55)

Age	−0.0143^*∗∗∗*^	−0.0077^*∗*^
	(−16.64)	(−1.89)

KHROA		0.0945^*∗∗∗*^
		(2.91)

KHAge		0.0056
		(1.24)

Constant	0.1005^*∗∗∗*^	0.0982^*∗∗∗*^
	(28.68)	(2.97)

Year	Yes	Yes

Industry	Yes	Yes
*N*	28391	1089
*R* ^2^	0.1508	0.2101

*Note. ∗∗∗*, *∗∗*, and *∗*indicate that the test coefficients are significant at the 1%, 5%, and 10% levels, respectively, and in parentheses, it displays the value *t*.

**Table 7:** Regression results of the adjustment effect of monetary policy and industry competitiveness.

	(1)	(2)
	Invest	Invest
CashFlow	0.0899^*∗∗∗*^	0.0736^*∗∗∗*^
	(2.74)	(2.61)

Risk	0.0286	0.0371
	(1.16)	(1.57)

Risk*∗*CashFlow	1.4678^*∗*^	1.4242^*∗∗∗*^
	(1.70)	(2.75)

Risk*∗*CashFlow*∗*MP	−0.2433^*∗*^	
	(−1.69)	

MP	0.0008	
	(1.15)	

Risk*∗*CashFlow*∗*HHI		−6.6113^*∗*^
		(−1.67)

HHI		0.0248
		(1.25)

Hold	0.0235^*∗∗∗*^	0.0204^*∗∗*^
	(2.60)	(2.07)

Std	0.0394^*∗∗∗*^	0.0094^*∗∗∗*^
	(4.38)	(3.10)

Msh	0.0314^*∗∗∗*^	0.0351^*∗∗∗*^
	(4.74)	(4.79)

ROA	0.0536	0.0513^*∗*^
	(1.45)	(1.94)

Growth	−0.0082^*∗*^	−0.0021
	(−1.68)	(−0.57)

Age	−0.0094^*∗∗*^	−0.0077^*∗*^
	(−2.34)	(−1.90)

KHROA	0.1127^*∗∗∗*^	0.0989^*∗∗∗*^
	(3.29)	(3.00)

KHAge	0.0031	0.0058
	(0.70)	(1.29)

Constant	0.0840^*∗∗∗*^	0.0941^*∗∗∗*^
	(2.86)	(2.84)

Year	Yes	Yes
Industry	Yes	Yes
*N*	1089	1088
*R* ^2^	0.2203	0.2101

*Note. ∗∗∗*, *∗∗*, and *∗* indicate that the test coefficients are significant at the 1%, 5%, and 10% levels, respectively, and in parentheses, it displays the value *t*.

The article "Empirical Analysis of Customer Risk and Corporate Financing Constraints Based on Supply Chain Networks" was published in 2022. Journal: Comput Intell Neurosci.

**Table 8:** Summary table of robustness test results 1.

	(1)	(2)
	Invest	Invest
CashFlow	0.0734^*∗∗∗*^	0.0649^*∗∗*^
	(2.77)	(2.27)

Risk	0.0338	0.0296
	(1.58)	(1.23)

risk*∗*CashFlow	0.9821^*∗∗*^	0.8667^*∗∗*^
	(2.49)	(2.18)

Hold	0.0198^*∗∗*^	0.0172^*∗*^
	(2.01)	(1.69)

Std	0.0097^*∗∗∗*^	0.0107^*∗∗∗*^
	(3.32)	(3.59)

Msh	0.0351^*∗∗∗*^	0.0301^*∗∗∗*^
	(4.80)	(3.71)

ROA	0.0481^*∗*^	0.0617^*∗∗*^
	(1.87)	(2.25)

Growth	−0.0020	−0.0035
	(−0.55)	(−0.94)

Age	−0.0078^*∗*^	−0.0073^*∗*^
	(−1.92)	(−1.77)

Size		0.0003
		(0.22)

Dual		0.0100^*∗∗∗*^
		(2.75)

Board		−0.0017
		(−0.51)

PPE		−0.0020
		(−0.21)

KHROA	0.0877^*∗∗∗*^	0.0852^*∗∗*^
	(2.66)	(2.56)

KHAge	0.0050	0.0073
	(1.11)	(1.60)

Constant	0.0997^*∗∗∗*^	0.0889^*∗∗*^
	(3.02)	(2.05)

Year	Yes	Yes
Industry	Yes	Yes
*N*	1088	1062
*R* ^2^	0.2089	0.2146

*Note. ∗∗∗*, *∗∗*, and *∗*indicate that the test coefficients are significant at the 1%, 5%, and 10% levels, respectively, and in parentheses, it displays the value *t*.

**Table 9:** Summary table of robustness test 2.

	(1)	(2)
	Invest	Invest
CashFlow	0.0260	0.0620
	(0.69)	(1.40)

Risk	0.0119	0.0805^*∗∗*^
	(0.42)	(2.49)

Risk*∗*CashFlow	1.5114^*∗∗∗*^	0.9565^*∗*^
	(3.06)	(1.90)

Hold	0.0142	0.0042
	(1.15)	(0.25)

Std	0.0099^*∗∗∗*^	0.0092^*∗∗∗*^
	(3.19)	(2.63)

Msh	0.0401^*∗∗∗*^	0.0273^*∗∗*^
	(4.80)	(2.49)

ROA	0.0252	−0.0070
	(0.66)	(−0.11)

Growth	−0.0081	0.0010
	(−1.51)	(0.19)

Age	−0.0081	−0.0070
	(−1.60)	(−1.18)

KHROA	0.0550	0.0435
	(1.38)	(0.84)

KHAge	0.0112^*∗∗*^	−0.0023
	(2.04)	(−0.33)

Constant	0.0169	0.1110^*∗*^
	(0.56)	(1.93)

Year	Yes	Yes
Industry	Yes	Yes
*N*	694	439
*R* ^2^	0.1644	0.2015

*Note. ∗∗∗*, *∗∗*, and *∗*indicate that the test coefficients are significant at the 1%, 5%, and 10% levels, respectively, and in parentheses, it displays the value *t*.

**Table 10:** Summary table of robustness test results 3.

	(1)
	FC
CRT	0.0103^*∗∗*^
	(2.21)

CashFlow	0.0303
	(1.30)

Age	0.0811^*∗∗∗*^
	(19.69)

Size	0.0023
	(1.57)

PPE	0.0004
	(0.04)

Lev	0.0044
	(0.48)

Hold	−0.0371^*∗∗∗*^
	(−3.70)

Msh	−0.0183^*∗∗*^
	(−2.32)

ROA	0.0495^*∗*^
	(1.66)

Growth	0.0039
	(1.22)

Dual	−0.0203^*∗∗∗*^
	(−5.64)

KHROA	0.0551
	(1.64)

KHAge	0.0042
	(0.95)

Constant	1.0518^*∗∗∗*^
	(18.96)

Year	Yes
Industry	Yes
*N*	1032
*R* ^2^	0.5525

*Note. ∗∗∗*, *∗∗*, and *∗*indicate that the test coefficients are significant at the 1%, 5%, and 10% levels, respectively, and in parentheses, it displays the value *t*.

**Table 11:** Two-stage least squares regression results 1.

	(1)	(2)	(3)
	Risk	Risk*∗*CashFlow	Invest
L.risk	0.8147^*∗∗∗*^	−0.0002	
	(13.90)	(-0.05)	

L.risk*∗*CashFlow	−1.1793	0.6611^*∗∗∗*^	
	(−1.55)	(3.35)	

Risk			0.0847
			(1.42)

Risk*∗*CashFlow			1.6162^*∗∗*^
			(2.52)

Control	Yes	Yes	Yes

Constant	0.0404^*∗∗*^	0.0016	0.1400^*∗∗∗*^
	(2.21)	(1.17)	(4.35)

Year	Yes	Yes	Yes
Industry	Yes	Yes	Yes
*N*	485	485	485
*R* ^2^	0.6173	0.6185	0.2351

*Note. ∗∗∗*, *∗∗*, and *∗*indicate that the test coefficients are significant at the 1%, 5%, and 10% levels, respectively, and in parentheses, it displays the value *t*.

The article "Empirical Analysis of Customer Risk and Corporate Financing Constraints Based on Supply Chain Networks" was published in 2022. Journal: Comput Intell Neurosci.

**Table 12:** Two-stage least squares regression results 2.

	(1)	(2)	(3)
	Risk	Risk*∗*CashFlow	Invest
OC	0.0502^*∗∗*^	−0.0036^*∗*^	
	(2.43)	(−1.82)	

OC*∗*CashFlow	−0.0781	0.0591^*∗∗∗*^	
	(−1.63)	(6.40)	

Risk			0.1053
			(0.33)

Risk*∗*CashFlow			2.4237^*∗∗∗*^
			(3.39)

Control	Yes	Yes	Yes

Constant	0.0973^*∗∗*^	0.0001	0.0344
	(2.12)	(0.02)	(0.74)

Year	Yes	Yes	Yes
Industry	Yes	Yes	Yes
*N*	855	855	855
*R* ^2^	0.0732	0.2716	0.1756

*Note. ∗∗∗*, *∗∗*, and *∗* indicate that the test coefficients are significant at the 1%, 5%, and 10% levels, respectively, and in parentheses, it displays the value *t*.

## Data Availability

The data used to support the findings of this study are included within the article.
